The article "Association of CYP2A6*4 with Susceptibility of Lung Cancer: A Meta-Analysis" was retracted in 2016. Reasons: compromised peer review; false authorship; ethical violations by an author.

# Association of CYP2A6*4 with Susceptibility of Lung Cancer: A Meta-Analysis

**DOI:** 10.1371/journal.pone.0059556

**Published:** 2013-04-09

**Authors:** Lishan Wang

**Affiliations:** 1 Bio-X Institutes and Affiliated Changning Mental Health Center, Key Laboratory for the Genetics of Developmental and Neuropsychiatric Disorders (Ministry of Education), Shanghai Jiao Tong University, Shanghai, P.R. China; 2 FengHe (ShangHai) Information Technology Co., Ltd, Minhang District, Shanghai, China; MOE Key Laboratory of Environment and Health, School of Public Health, Tongji Medical College, Huazhong University of Science and Technology, China

## Abstract

**Objectives:**

To assess the association between the variant of Cytochrome P450 2A6 whole gene deletion (CYP2A6*4) polymorphism and risk of lung cancer.

**Methods:**

Two investigators independently searched the PubMed, Elsevier, EMBASE, Web of Science, Wiley Online Library and Chinese National Knowledge Infrastructure (CNKI). Pooled odds ratios (ORs) and 95% confidence intervals (95% CIs) for CYP2A6*4 and lung cancer were calculated in a fixed-effects model (the Mantel-Haenszel method) and a random-effects model (the DerSimonian and Laird method) when appropriate.

**Results:**

This meta-analysis included seven eligible studies, which included 2524 lung cancer cases and 2258 controls (cancer–free). Overall, CYP2A6*4 was associated with the risk of lung cancer (allele*4 vs. allele non-*4, pooled OR  = 0.826, 95% CI  = 0.725−0.941, P-value  = 0.004). When stratifying for population, significant association was observed in Asian (additive model, pooled OR  = 0.794, 95% CI  = 0.694−0.909, P-value  = 0.001; dominant model, pooled OR  = 0.827, 95% CI  = 0.709−0.965, P-value  = 0.016; recessive model (pooled OR  = 0.444, 95% CI  = 0.293−0.675, P-value <0.0001). In the overall analysis, a comparably significant decrease in the frequency of *4/*4 genotype was detected between cases and controls in Asian while no *4/*4 genotype was detected in Caucasian in collected data.

**Conclusion:**

This meta-analysis suggests that the CYP2A6*4 polymorphism is associated with susceptibility of lung cancer in Asian. The whole gene deletion of *CYP2A6* may decrease the risk of lung cancer in Asian samples.

## Introduction

Lung cancer is the most common cancer in the world, representing approximately 12% of all new cancer cases, with over 1 million deaths annually, which is the leading cause of cancer death [1]. It is well-known that smoking is a major cause of lung cancer. It is reported that environmental tobacco smoke increases the risk of lung cancer in nonsmokers by approximately 20–50% [2].

Tobacco carcinogens are the most significant factors for smoking induced cancers. To exert their effects, most tobacco carcinogens require metabolic activation, which is generally carried out by cytochrome P450 (CYP) enzymes. Short-lived electrophile agents produced in metabolic activation process react with DNA, thus causing DNA damage and inducing tumors. Such process, mostly, only happen in tissues where it is generated. Therefore, tissue-specific metabolic activation is of vital importance for tissue susceptibility to carcinogen-induced tumors. Among tobacco's potent carcinogens, tobacco-specific nitrosamines (TSNA) and other nitrosamines are activated by CYP2A enzymes, nicotine is also metabolized by CYP2A enzymes [3]–[4].

The article "Association of CYP2A6*4 with Susceptibility of Lung Cancer: A Meta-Analysis" was retracted in 2016. Reasons: compromised peer review; false authorship; ethical violations by an author.

There are three CYP2A genes in humans (*CYP2A6*, *CYP2A7* and *CYP2A13*) and one pseudogene (*CYP2A18*)[5], but there is no catalytic activity shown for *CYP2A7* so far. *CYP2A6* expression is mainly found in the liver, but its protein or mRNA is also expressed in other tissues such as nasal epithelium, trachea, lung and esophagus [6]–[7]. There are 31 numbered CYP2A6 allelic variants identified to date, however, not all have been functionally characterized. The different alleles are described at the Human CYP Allele Nomenclature Committee Homepage (www.cypalleles.ki.se/cyp2a6.htm). CYP2A6*4 presents a gene deletion that accounts for the majority of poor metabolizer individuals (PM) in Asian populations, and various alleles have been described [8]–[9]. Currently, three deletion variants are known for CYP2A6*4. CYP2A6*4A lacks the 3′-UTR of the CYP2A7 gene and the whole CYP2A6 gene is deleted and an unequal crossover junction is located in the 3′-UTR. CYP2A6*4B has a normal CYP2A7 gene, while the whole CYP2A6 gene is deleted. In CYP2A6*4D, an unequal crossover junction is located at the end of the CYP2A7 gene in either exon 8 or 9 and the whole CYP2A6 gene is deleted. Formerly, a CYP2A6*4C allele is recognized, but subsequent observations reveal that this allele is the same as the CYP2A6*4A allele. Because all these variants result in a whole gene deletion of CYP2A6, most studies do not discriminate between the variants and the term ‘CYP2A6*4’ is designated to all deletions [8]–[9].

During this decade, a number of studies have assessed the association between CYP2A6*4 polymorphism and risk of lung cancer in different populations; however, the results are inconsistent and inconclusive [[10]–[11]]. Dif­ferent methodologies have been used, however, in particular, most of the studies use a small sample size and it is therefore not surprising that there has been a lack of replication in the various studies. As meta-analysis is an effective way to increase the statistical power by pooling all the available data together and analyzing with a large dataset, in which all the published case-control studies are processed to confirm whether the CYP2A6*4 polymorphism is associated with susceptibility of lung cancer.

The article "Association of CYP2A6*4 with Susceptibility of Lung Cancer: A Meta-Analysis" was retracted in 2016. Reasons: compromised peer review; false authorship; ethical violations by an author.

## Materials and Methods

### Literature search

The PubMed, Elsevier, EMBASE, Web of Science, Wiley Online Library and Chinese National Knowledge Infrastructure (CNKI) for all articles were searched with the following search terms: (‘*CYP2A6*’ OR ‘Cytochrome P450 2A6’) AND (‘lung cancer’). The date of the last search was Sep 20, 2012. Publication date and publication language were not restricted in our search. Reference lists were examined manually to further identify potentially relevant studies. Unpublished reports were not considered. If more than one article was published by the same author using the same case series, we selected the study where the most individuals were investigated.

### Inclusion and exclusion criteria

Abstracts of all citations and retrieved studies were reviewed. Studies meeting the following criteria were included: (1) Using a case – control design; (2) Detecting the relationship between variant CYP2A6*4 and lung cancer; (3) Providing available genotype data of CYP2A6*4; (4) Control group is cancer-free. Studies were excluded if one of the following factors existed: (1) the design is based on family or sibling pairs or case-only; (2) the genotype frequency of CYP2A6*4 is not reported; or (3) there is insufficient information for extraction of data.

### Data extraction

All data were extracted independently by two reviewers (XXX and XXX) according to the inclusion criteria listed above. Disagreements were resolved by discussion between the two reviewers. The following characteristics were collected from each study: first author, year of publication, country of sample, ethnicity, number of cases and controls, main background of samples, matching criteria, and genotyping methods (Table 1).

**Table 1:** Characteristics of studies included in the meta-analysis.

Author	Year	Country	Population	No.(cases /controls)	Gender	Smoking status	Matchingcriteria	Genotypingmethods	Ref.
Miyamoto	1999	Japan	Asian	246/201	Mixed	Mixed	Age, sex, race	PCR-RFLP	[^15^]
Loriot	2001	France	Caucasian	244/250	Male	All smokers	Age, sex, race	PCR-RFLP	[^16^]
Tan	2001	China	Asian	151/326	Mixed	Mixed	Age, sex, race	PCR-RFLP	[^17^]
Fujieda	2004	Japan	Asian	1094/611	Male	All smokers	Age, sex, race	PCR-RFLP	[^18^]
Gu	2005	China	Asian	180/224	Mixed	Mixed	Age, sex, race	PCR-RFLP	[^19^]
Tamaki	2011	Japan	Asian	192/203	Mixed	Mixed	Age, sex, race	PCR-RFLP	[^20^]
Wassenaar	2011	Canada	Caucasian	417/443	Mixed	All smokers	Age, sex, race	PCR-RFLP	[^21^]

PCR-RFLP: Polymerase chain reaction-restriction fragment length polymorphism.

The article "Association of CYP2A6*4 with Susceptibility of Lung Cancer: A Meta-Analysis" was retracted in 2016. Reasons: compromised peer review; false authorship; ethical violations by an author.

### Statistical analysis

The statistical analysis was conducted using STATA 11.0 (Stata Corp LP, College Station, TX, United States); P-value <0.05 was considered statistically significant. Hardy Weinberg Equilibrium (HWE) in the controls was tested by the chi-square test for goodness of fit, and a P –value <0.05 was considered as significant disequilib­rium. Pooled ORs were calculated for allele frequency comparison (*4 vs. non-*4), dominant model (*4/*4+*4/non-*4 vs. non-*4/non-*4), and recessive model ((*4/*4 vs.*4/non-*4 +non-*4/non-*4)), respectively. The significance of pooled ORs was determined by Z-test and P-value <0.05 was considered statistically significant.

The OR and 95% CI were estimated for each study in a random-effects model or a fixed-effects model. Heterogeneity among studies was examined with the χ^2^ -based Q testing and *I^2^* statistics [12]. P-value <0.1 was consid­ered significant for the χ^2^-based Q testing and I^2^ was interpreted as the proportion of total variation contributed by between-study variation. If there was a significant het­erogeneity (P-value <0.1), a random-effects model (the DerSimonian and Laird method) was selected to pool the data. If not, a fixed-effects model (the Mantel-Haenszel method) was selected to pool the data. Heterogeneity was also quantified using the *I^2^* metric (*I^2^*<25%, no heterogeneity; *I^2^*  = 25–50%, moderate heterogeneity; *I^2^*>50%, large or extreme heterogeneity) [25]. Publication bias was examined with funnel plots and with the Egger's tests [13]–[14]. If there is evidence of publication bias, the funnel plot is noticeably asymmetric. For the Egger's tests, the significance level was set at 0.05.

## Results

### Study Characteristics

A total of 52 papers were retrieved after the first search. After our selection, 7 case-control studies including 2524 lung cancer cases and 2258 controls fulfilled the inclusion criteria [10]–[11]. The qualities of the studies were considered acceptable for our meta-analysis. HWE were calculated for all seven publications and found that only Tamaki's study was inconsistent with Hardy-Weinberg disequilibrium (P-value  = 0.042). The flow chart of selection of studies and reasons for exclusion is presented in Figure 1. Studies had been carried out in Japan, France, China and Canada. Five studies [10], [15]–[16] used Asian samples while two studies [17] , [11] used Caucasian samples. Characteristics of studies included in the meta-analysis are presented in Tables 1 and 2.

**Figure 1:** Flow chart of selection of studies and specific reasons for exclusion from the meta-analysis.

The article "Association of CYP2A6*4 with Susceptibility of Lung Cancer: A Meta-Analysis" was retracted in 2016. Reasons: compromised peer review; false authorship; ethical violations by an author.

**Table 2:** Genotype frequencies of CYP2A6*4 in studies included in the meta-analysis.

Author	Year	Case genotype^a^			Control genotype^b^			HWE^c^	Ref.
		*4/*4	*4/non-*4	non-*4/non-*4	*4/*4	*4/non-*4	non-*4/non-*4		
Miyamoto	1999	5	48	193	9	60	132	0.3507	[^15^]
Loriot	2001	0	24	220	0	19	231	1.0000	[^16^]
Tan	2001	1	38	112	5	46	275	0.0735	[^17^]
Fujieda	2004	25	301	768	28	186	397	0.3082	[^18^]
Gu	2005	0	23	157	1	30	193	1.0000	[^19^]
Tamaki	2011	7	63	122	19	66	118	0.042	[^20^]
Wassenaar	2011	0	6	411	0	0	443	1.0000	[^21^]

a Absolute number of patients; ^b^ Absolute number of controls; ^c^ HWE: Hardy-Weinberg equilibrium, which was evaluated using the goodness-of-fit chi-square test. P < 0.05 was considered representative of a departure from HWE.

### Evaluation of CYP2A6*4 and association with lung cancer

There were seven case-control studies [10]–[11] which had been performed to study the CYP2A6*4 poly­morphism and lung cancer risk. Results of the meta-analysis are shown in Table 3. Results showed that there was a significant association be­tween CYP2A6*4 polymorphism and lung cancer risk (additive model, pooled OR  = 0.826, 95% CI  = 0.725–0.941, P-value  = 0.004). But no significant association was observed under dominant model (pooled OR  = 0.867, 95% CI  = 0.747–1.006, P-value  = 0.06).

**Table 3:** Pooled odds ratio for CYP2A6*4 in meta-analyses.

Population	Genetic Model	Pooled OR(95% CI)	P-value^a^	P-value^b^(Publication bias)	P-value^c^(heterogeneity)	I^2^
All	Additive	0.826(0.725–0.941)	0.004	0.177	0.002	71.4%
	Dominant	0.867(0.747–1.006)	0.06	0.211	0.001	72.9%
Asian	Additive	0.794(0.694–0.909)	0.001	0.622	0.005	73.0%
		0.737(0.640–0.848)^d^	<0.0001	0.800	0.370	4.5%
	Dominant	0.827(0.709–0.965)	0.016	0.791	0.002	75.7%
		0.751(0.637–0.884)^e^	0.001	0.804	0.324	13.7%
	Recessive	0.444(0.293–0.675)	<0.0001	0.486	0.990	0.0%
Caucasian	Additive	1.640(0.919–2.927)	0.094	–	0.105	62.0%
	Dominant	1.674(0.927–3.024)	0.088	–	0.106	61.8%

a Random-effects model was used when the p-value for heterogeneity test<0.10, otherwise the fixed-effect model was used. ^b^ Egger's test to evaluate publication bias. P –value <0.05 is considered statistically significant. ^c^ P-value <0.1 is considered statistically significant for Q statistics. ^d and e^ The results of Asian samples after exclusion of Tan's study. OR: Odds ratio; CI: confidence interval.

When studies were divided according to the population, the results indicated that significant associations were observed in Asian samples under all models (additive model, pooled OR  = 0.794, 95% CI  = 0.694–0.909, P-value  = 0.001; dominant model, pooled OR  = 0.827, 95% CI  = 0.709–0.965, P-value  = 0.016; recessive model (pooled OR  = 0.444, 95% CI  = 0.293–0.675, P-value <0.0001). Reversely, no significant associations were observed in Caucasian samples under any model (allele, pooled OR  = 1.640, 95% CI  = 0.919–2.927, P-value  = 0.094; dominant model, pooled OR  = 1.674, 95% CI  = 0.927–3.024, P-value  = 0.088; recessive model was not available as no *4/*4 genotype was observed in Caucasian samples). Results of the meta-analysis are shown in Table 3 and Figure 2.

The article "Association of CYP2A6*4 with Susceptibility of Lung Cancer: A Meta-Analysis" was retracted in 2016. Reasons: compromised peer review; false authorship; ethical violations by an author.

**Figure 2:** Forest plots of all studies and studies with Asian samples under different genetic models. **a**. All studies (Additive model). **b**. Studies with Asian samples (Additive model). **c**. Studies with Asian samples (Recessive model). **d**. Studies with Asian samples (Dominant model).

### Sensitivity analysis

The influence of a single study on the overall meta-analysis estimate was investigated by omitting one study at a time, and the omission of any study made no significant difference, indicating that our results were statistically reliable.

### Evaluation of heterogeneity and publication bias

For all studies, statistically significant heterogeneity was observed (P-values by χ2-based Q testing <0.1 and *I^2^* >50%). Then subgroup analysis was carried out. Studies were divided according to the population. For Caucasian, no statistically significant heterogeneity was observed under either additive model (*4 vs. non-*4, P-value  = 0.105) or dominant model (*4/*4+*4/non-*4 vs. non-*4/non-*4, P-value  = 0.106). For Asian, no statistically significant heterogeneity was observed under recessive model (*4/*4 vs. *4/non-*4 + non-*4/non-*4, P-value  = 0.990, I2 = 0), but significant heterogeneity was still observed under both additive model (*4 vs. non-*4, P-value  = 0.005) and dominant model (*4/*4+*4/non-*4 vs. non-*4/non-*4, P-value  =  0.002). However, when Tan's study was excluded, no statistically significant heterogeneity was observed anymore under either additive model (*4 vs. non-*4, P-value  = 0.370, I2  = 4.5%) or dominant model (*4/*4+*4/non-*4 vs. non-*4/non-*4, P-value  = 0.324, I2  = 13.7%). Funnel plot and Egger's test were performed to assess the publication bias of the literature. No publication bias was observed (all P-value of Egger's test >0.05) and symmetrical funnel plots were obtained. Results of heterogeneity and publication bias are shown in Table 2.

## Discussion

As previous research reported, allele frequency of CYP2A6*4 differed significantly between Asian and non-Asian. CYP2A6*4 is more prevalent among Japanese individuals, with an allele frequency of approximately 0.200[18],[19]–[20]. The frequency is also relatively high among Koreans and Thais (0.110 and 0.140, respectively)[20],[21]. Among Brazilians, French individuals and Canadians, the frequency is 0.010 or lower [22],[23],[24]. The data from this meta-analysis showed a significant decrease of genotype frequency of *4/*4 for the CYP2A6*4 polymorphism in patients with lung cancer than controls in Asian, which suggest that genotype *4/*4 of CYP2A6*4 may decrease the risk of lung cancer in Asian. Therefore, significant results were only discovered in Asian, but not non-Asian population, which may be caused by low frequency of CYP2A6*4 polymorphism. In addition, it is reported that the plasma concentration of cotinine, a major metabolite of nicotine, is considerably higher in carriers of wild-type alleles of *CYP2A6* than that in carriers of null or reduced-function alleles of *CYP2A6*, raising the possibility that cotinine plays an important role in the development of lung cancer [25]. It is also reported that lung tumorigenesis can be promoted by anti-apoptotic effects of cotinine through activation of PI3K/Akt pathway, which is mediated by *CYP2A6* [26]. These previous findings support our results and give us possible explanation to the mechanism.

The article "Association of CYP2A6*4 with Susceptibility of Lung Cancer: A Meta-Analysis" was retracted in 2016. Reasons: compromised peer review; false authorship; ethical violations by an author.

The degree of heterogeneity is one of the major concerns in a sound meta-analysis because non-homogeneous data are liable to result in misleading results. In the present study, the *Q* testing and *I*^2^ statistics were carried out to test the significance of heterogeneity. For all studies, there existed significant heterogeneity. So subgroup analysis was made according to the ethnicity of samples. No significant heterogeneity was observed in Caucasian under any model or in Asian under recessive model. But significant heterogeneity existed in Asian under the other two models, and Tan's study was found to be responsible for heterogeneity. After removing this study, no significant heterogeneity was observed (both P-value of Q testing>0.1, shown in Table 2). Moreover, we performed a sensitivity analysis by removing one study each time and rerunning the model to determine the effect on each overall estimate. The estimates changed little, which implied that our results were statistically reliable.

However, there are still some limitations in this meta-analysis. (1) In seven studies included for our analysis, only two of them are Caucasian samples; (2) The samples from 4 countries and controls are not uniform; (3) CYP2A6*4 is related with smoking, but the smoking status of samples is not uniform in our study. Thus, results should be interpreted with caution; (4) Number of studies and number of subjects in the studies included in the meta-analysis are still small; and (5) Meta-analysis is a retrospective research that is subject to some methodological limitations. In order to minimize the bias, we used explicit methods for study selection, data extraction and data analysis. Nevertheless, our results should be interpreted with caution.

The article "Association of CYP2A6*4 with Susceptibility of Lung Cancer: A Meta-Analysis" was retracted in 2016. Reasons: compromised peer review; false authorship; ethical violations by an author.

This meta-analysis suggests that the CYP2A6*4 polymorphism is associated with susceptibility of lung cancer in Asian and the whole gene deletion of *CYP2A6* may decrease the risk of lung cancer. The pooled ORs in this study suggest that *4/*4 genotype has a modest but definite genetic effect in Asian. Larger and well-designed studies based on different ethnic groups are needed to confirm our results.

## Supporting Information

Checklist S1 **PRISMA Checklist**.
(DOC)
